RETRACTED

# A Retrospective Case-Control Study on Late Failure of Arteriovenous Fistula in Hemodialysis Patients and Prediction of Risk Factors

**DOI:** 10.1155/2022/8110289

**Published:** 2022-03-08

**Authors:** Liang Ge, Yu Fang, Shaofeng Rao

**Affiliations:** Department of Nephrology, Xianning Central Hospital, Xianning City 437000, China

## Abstract

**Objective:**

A retrospective case-control study was conducted to explore the risk factors of late failure of arteriovenous fistula in hemodialysis patients.

**Methods:**

A total of 95 hemodialysis patients treated in our hospital from January 2018 to January 2021 were included. The HE staining results of late failure of arteriovenous fistula in hemodialysis patients were observed. The general data and laboratory indexes of the patients were recorded by using a questionnaire survey, hospital case system, and hemodialysis record. According to the functional status of internal fistula, the patients were divided into two groups: failure group (*n* = 35) and patency group (*n* = 60). SPSS22.0 software was employed for statistical analysis, and the relevant data of the two groups were compared. The independent sample *t*-test was employed for the comparison of variance between groups, and the *χ*^2^ test was employed for counting data. Logistic multivariate regression was employed to analyze the risk factors of late loss of power in autologous arteriovenous fistula (AVF).

**Results:**

(1) Late failure of arteriovenous fistula in hemodialysis patients: the results of HE staining showed the following: (1) histological changes of venous intima: 100% of the patients had varying degrees of intimal hyperplasia, mainly eccentric hyperplasia, resulting in luminal stenosis, and annular uniform intimal hyperplasia in some patients, and (2) histological changes of venous media: 81.6% of the patients had venous media lesions, which were mainly in two cases; one was media smooth muscle hyperplasia with fibrous tissue hyperplasia, and the other was smooth muscle compression when intimal hyperplasia was serious, resulting in smooth muscle fiber rupture, disarrangement, focal necrosis, atrophy, and thinning, and some smooth muscle stroma showed vitreous degeneration and myxoid degeneration. A few cases showed multifocal neutrophil, lymphocyte, and plasma cell infiltration. (2) First of all, we surveyed the general data, and there were significant differences in age, history of diabetes, history of hypertension, and uric acid nephropathy (*P* < 0.05). There was no significant difference in sex, body mass index, smoking history, polycystic kidney disease, chronic glomerulonephritis, and obstructive nephropathy between the two groups (*P* > 0.05). Secondly, we compared the levels of hemoglobin, eosinophils, platelet count, and hematocrit. The levels of hemoglobin, eosinophils, and hematocrit in the failure group were higher, and the platelet count was lower compared to that of the unobstructed group (*P* < 0.05). Furthermore, the calcium and phosphorus product and the level of C-reactive protein (CRP) in the failure group were higher, while the levels of fibrinogen and INR in the unobstructed group were lower. The levels of plasma protein, alkaline phosphatase, and cholesterol were higher in the failure group, while the level of triglyceride was lower in the failure group (*P* < 0.05). Finally, logistic regression analysis showed that age, hemoglobin, hematocrit, and calcium-phosphorus product were the risk factors for late failure of arteriovenous fistula in hemodialysis patients (*P* < 0.05). There exhibited no significant correlation between diabetes, hypertension, uric acid nephropathy, eosinophil, CRP, fibrinogen, INR, plasma protein, alkaline phosphatase, cholesterol, triglyceride, and late failure of arteriovenous fistula in hemodialysis patients.

RETRACTED

**Conclusion:**

Age, hemoglobin, hematocrit, and calcium-phosphorus product are independent risk factors for late failure of arteriovenous fistula in hemodialysis patients. The hemoglobin, eosinophil, platelet count, and hematocele in hemodialysis patients with late failure of arteriovenous fistula were higher. The indexes related to biochemistry, blood coagulation, and nutrition were significantly different from those without late failure of arteriovenous fistula. Thus, the risk of late failure of arteriovenous fistula can be predicted.

## 1. Introduction

The ultimate outcome of continuous progression of chronic kidney disease (CKD) is end-stage renal disease (ESRD). The global incidence of CKD is on the rise, with an estimated prevalence rate of 8%-16%, which has a significant impact on the global disease burden and has become a public health issue [1]. In March 2015, a study by Dr. Hoeerger showed that the incidence of CKD will increase sharply in the next 20 years [2]. The epidemiological survey of CKD in China indicates that the prevalence rate of CKD in Chinese adults is 10.8%, of which ESRD patients account for 1.7-5.8% [3]. Renal replacement therapy for ESRD patients mainly includes hemodialysis (HD), peritoneal dialysis (PD), and renal transplantation. However, the most effective alternative therapy is still hemodialysis. According to statistics, about 1.5 million ESRD patients worldwide use hemodialysis as a renal replacement therapy [4]. Vascular access is a prerequisite for hemodialysis, and the quality of vascular access directly affects the dialysis and quality of life of patients [5].

RETRACTED

Autologous arteriovenous fistula (AVF) is to anastomose the artery and vein subcutaneously by end-to-side or end-to-end [6]. After a period of maturity, the vein wall is arterialized, the vein mixes part of the arterial blood, and the blood flow increases. The pressure increases to achieve the blood flow needed for dialysis. Arteriovenous fistula mainly includes AVF, artificial vascular graft arteriovenous fistula, and allograft internal fistula [6]. The NKF-K/DOQI working group suggests that AVF should be employed as far as possible. Because of its few complications, high patency rate, convenient operation, and low cost, it is helpful to improve the quality of life and survival rate of patients. In view of many advantages, AVF is the most commonly employed method of internal fistula [6]. However, due to poor vascular conditions, it is feasible to graft arteriovenous fistula with artificial blood vessels if it is not suitable for autogenous arteriovenous fistula. If all kinds of arteriovenous fistula cannot be employed, central venous catheterization can only be chosen [6]. A study unveiled that among maintenance hemodialysis patients, 80.33% of patients with nontunnel and nonpolyester cannula constitutes 8.19% for the first dialysis, 9.84% for a tunnel catheter with polyester sheath, and 1.64% for arteriovenous puncture, and 87.60% of patients with AVF and 12.40% of patients with a tunnel catheter with polyester sheath accounted for 87.60% and 12.40%, respectively, in the later stage of maintenance hemodialysis [7]. Therefore, AVF is the most important vascular pathway for hemodialysis patients, and it is an important channel for maintenance hemodialysis patients to maintain life. Whether it is unobstructed or not directly affects the quality of life and survival rate of hemodialysis patients. Thus, this paper surveyed the important risk factors for late AVF failure in patients with MHD in our hospital and actively took relevant intervention measures to prolong their service life for different patients.

## 2. Patients and Methods

### 2.1. Participant Information

A total of 95 hemodialysis patients treated in our hospital from January 2018 to January 2021 were enrolled. According to the functional status of internal fistula, the patients were assigned into two groups: failure group (*n* = 35, first loss of work) and patency group (*n* = 60). The inclusion criteria were as follows: (1) age > 18 years old; (2) end-to-side anastomosis between the cephalic vein and radial artery in internal arteriovenous fistula; (3) mature arteriovenous fistula, more than one month; (4) hemodialysis three times a week; and (5) single upper arm fistulotomy for the first time. Exclusion criteria were as follows: (1) internal venous fistula in external hospital, (2) hemodialysis using a vascular pathway other than autologous arterial fistula, and (3) blockage of internal fistula caused by excessive compression. Criteria for judging the failure of internal arteriovenous fistula [8] were as follows: (1) doctors touched the pulsation or tremor of internal arteriovenous fistula, and no vascular murmur was found in auscultation; (2) the extracorporeal circulation line twitched during dialysis, and the blood flow was insufficient; (3) the epidermis temperature of internal fistula was significantly lower than that before; (4) when necessary, color Doppler ultrasound was performed to check that there was no blood flow signal in the diastolic period of internal fistula, indicating that arteriovenous fistula was blocked and no collateral circulation was formed; and (5) the blood flow is lower than that of 180 ml/min, which cannot meet the needs of dialysis.

RETRACTED

### 2.2. Therapeutic Methods

A retrospective study was conducted, and 95 subjects were included. According to the functional status of internal fistula, the patients were divided into two groups: failure group (*n* = 35) and patency group (*n* = 60). All the subjects underwent forearm AVF (excluding nasopharynx operation) by the same professional doctor in our hospital, and the anastomosed vessels were the cephalic vein-radial artery. The way of anastomosis was end-to-side anastomosis. When AVF matured, hemodialysis was maintained in our hospital, the frequency of dialysis was 2-3 times per week, the time of dialysis was 3.5-4 hours per time, the blood flow was 200~300 ml/min during dialysis, and anticoagulant with unfractionated heparin was employed.

The processing flow of vascular tissue specimens: all specimens were stained with hematoxylin-eosin (HE). (1) 0.5-1% eosin alcohol solution: eosin Y powder (alcohol soluble) 10 g was added to 95% ethanol solution of 1000 ml, stirred, and fully dissolved, and 0.5 ml glacial acetic acid was added to speed up the dyeing process. (2) Hematoxylin dye solution: weigh hematoxylin 2 g, mix with anhydrous ethanol 250 ml, fully stir, and dissolve. 5 g aluminum potassium sulfate was mixed with distilled water 750 ml and stirred fully. Then, mix hematoxylin ethanol solution and aluminum potassium sulfate solution evenly, add 0.2 g sodium iodate and stir fully, place for 5 minutes, then add glycerol 50 ml and citric acid 0.3 g to shake for several minutes, incubate it overnight, and then use it. (3) 1% hydrochloric acid alcohol differentiation solution: take concentrated hydrochloric acid 10 ml and add 95% ethanol 990 ml. (4) Dyeing process: (1) to make paraffin sections: after the biopsy tissue was fixed, dehydrated, rendered transparent, impregnated, and embedded into wax blocks, the paraffin sections were thick sliced with a paraffin slicer, spread with a spreader, and baked at 70°C for 30 minutes. The quality of the early operation of paraffin tissue wax production has a great influence on the detection results of subsequent paraffin sections, which are fixed with 10% neutral formalin and correctly dehydrated, rendered transparent, impregnated, and embedded in time. It is the premise guarantee for the follow-up detection of paraffin sections to get correct results. (2) Dewaxing to water: the paraffin slices were soaked in xylene 3 times for 10 minutes each time. After removing xylene, the paraffin slices were soaked in anhydrous ethanol twice for 2 minutes each time, then washed in 95% alcohol and 85% alcohol for 2 minutes, then rinsed with flowing tap water for 1 minute, and finally soaked in distilled water for use. Whether the dewaxing is clean or not directly affects the quality of the subsequent dyeing. If the dewaxing is not clean, the slices are opaque after rinsing with tap water, with water droplets attached, and dyeing is not easy or uneven. (3) HE staining: the dewaxed and hydrated slices were immersed in hematoxylin dye solution for 10 minutes, rinsed with flowing tap water for 30 seconds, then differentiated with 1% hydrochloric acid ethanol differentiation solution for 10 seconds, rinsed with flowing tap water for 30 seconds, then soaked in warm water at 50°C for 5 minutes, then rinsed with distilled water for 1 minute, immersed in 95% ethanol for 1 minute, and finally dyed in eosin ethanol solution for 1 minute. The stained slices were soaked in 95% ethanol for 2 minutes and anhydrous ethanol for 2 minutes, then immersed in xylene solution for 5 minutes, wet sealed or dried from anhydrous ethanol, and dried directly with neutral gum. HE staining results: the nucleus in the section showed blue, while the cytoplasm, erythrocytes, collagen fibers, muscle fibers, connective tissue, and eosinophilic granules showed different shades of red. The sections stained with HE should be intact, wrinkle-free, knife-free, uniform in thickness, clear in nucleus and cytoplasm, moderate in red and blue color, transparent and clean, and beautiful in appearance.

RETRACTED

### 2.3. Observation Index

#### 2.3.1. General Information

The basic clinical data of sex, age, body mass index, primary disease, hypertension, diabetes, and smoking history of ESRD patients with AVF were collected.

#### 2.3.2. Serum Index

The biochemical and coagulation indexes such as hemoglobin (Hb), eosinophil (EOS), hematocrit (HCT), platelet (PLT), C-reactive protein (CRP), plasma albumin (Alb), triglyceride (TG), cholesterol (TC), prothrombin time (PT), international standardized ratio (INR), and fibrinogen were collected and analyzed.

### 2.4. Statistical Analysis

SPSS 22.0 statistical software was employed to analyze the data. The counting data is represented by *n* (%), and the continuous variable data is represented by $\bar{x}\pm s$. The counting data were analyzed by the *χ*^2^ test, and the measurement data in accordance with normal distribution were compared by the independent sample *t*-test. The logistic multivariate regression method was employed to analyze the risk factors for late AVF failure (*P* < 0.05). The difference was statistically significant.

## 3. Results

### 3.1. HE Staining Results of Late Failure of Arteriovenous Fistula in Hemodialysis Patients

(1) Histological changes of venous intima: 100% of the patients had varying degrees of intimal hyperplasia, mainly eccentric hyperplasia, resulting in intraluminal stenosis (Figure 1(a)), and annular homogeneous intimal hyperplasia in some patients (Figure 1(b)). Intimal hyperplasia was mainly characterized by the proliferation of smooth muscle cells and fibrous cells, most of which were accompanied by mucinous degeneration and vitreous degeneration, inflammatory cell infiltration, and scattered parenchyma vascular hyperplasia in some cases. (2) Histological changes of venous media: 81.6% of the patients had venous media lesions, mainly in two cases: one was media smooth muscle hyperplasia with fibrous tissue hyperplasia (Figure 1(c)) and the other was when intimal hyperplasia was severe. Smooth muscle compression results in smooth muscle fiber rupture, disarrangement, focal necrosis, atrophy, and thinning (Figure 1(d)). Some smooth muscle stroma showed vitreous degeneration and myxoid degeneration, and a few cases showed multifocal neutrophil, lymphocyte, and plasma cell infiltration.

### 3.2. Comparison of General Data

First of all, we elucidated the general data of the two groups, and there was significant differences in age, history of diabetes, history of hypertension, and uric acid nephropathy (*P* < 0.05). There exhibited no significant difference in sex, body mass index, smoking history, polycystic kidney disease, chronic glomerulonephritis, and obstructive nephropathy (*P* > 0.05). All the data results are indicated in Table 1.

### 3.3. Comparison of Hemoglobin, Eosinophil, Platelet Count, and Hematocrit

Secondly, we compared the levels of hemoglobin, eosinophils, platelet count, and hematocrit. The levels of hemoglobin, eosinophils, and hematocrit were higher, and the platelet count was lower in the failure group compared to the unobstructed group (*P* < 0.05). All the data results are indicated in Table 2.

RETRACTED

### 3.4. Comparison of Biochemical and Coagulation Indexes

Next, we compared the blood biochemical and coagulation indexes. The calcium and phosphorus product and CRP levels were higher, while the levels of fibrinogen and INR were lower in the failure group compared to the unobstructed group (*P* < 0.05). There was no significant difference in PT between the two groups. All the data results are indicated in Table 3.

### 3.5. Comparison of Nutrition-Related Indexes

Then, we compared the nutrition-related indexes. The levels of plasma protein, alkaline phosphatase, and cholesterol were higher, while the level of triglyceride in the failure group was lower compared to the patency group (*P* < 0.05). All the data results are indicated in Table 4.

### 3.6. Logistic Regression Analysis of Risk Factors for Late Failure of Arteriovenous Fistula in Hemodialysis Patients

Finally, we carried out logistic regression analysis on the risk factors for late failure of arteriovenous fistula in hemodialysis patients. The results showed that age, hemoglobin, hematocrit, and calcium-phosphorus product were the risk factors for late failure of arteriovenous fistula in hemodialysis patients (*P* < 0.05). There was no significant correlation between diabetes, hypertension, uric acid nephropathy, eosinophil, CRP, fibrinogen, INR, plasma protein, alkaline phosphatase, cholesterol, triglyceride, and late failure of arteriovenous fistula in hemodialysis patients. The results of all the data are indicated in Table 5.

## 4. Discussion

With the rapid development of the economy, the acceleration of the aging of the population, and the improvement of people's lifestyle, the prevalence of CKD is increasing, and the patients with CKD will eventually end with chronic renal failure, so the population of maintenance hemodialysis (MHD) is also expanding [2]. CKD patients often have no obvious symptoms in the early stage, so the diagnosis rate is low, but in the later stage, because of the high cost of treatment, it has become an important public health problem [9]. Among the three different renal replacement therapies, hemodialysis (HD) is the most important because of its higher dialysis adequacy and higher long-term survival rate than those of the peritoneal dialysis group [3]. In recent years, with the increase in the prevalence of CKD, the number of MHD patients indicates a rapid growth trend. The choice of a vascular pathway is very important for hemodialysis patients, which is an important life channel for maintenance hemodialysis patients [5]. AVF has become the first choice for patients with MHD because of its convenient use, few complications, and long-term durability. The functional state of arteriovenous fistula directly affects the dialysis efficiency and quality of life of uremic patients, so it is very important to study the risk factors of arteriovenous fistula blockage in patients with maintenance arteriovenous hemodialysis and to prevent arteriovenous fistula blockage [10, 11].

RETRACTED

AVF has become the preferred long-term vascular pathway at home and abroad because of its low risk of fatal infection, low all-cause mortality, convenient operation, few complications, repeated puncture, stable blood flow, long service life, and so on [12]. K-DOQI (the National Kidney Foundation Kidney-Dialysis Outcomes Quality Initiative), CPM (Clinical Performance Measures), and other studies also emphasized that autologous AVF is the first choice for hemodialysis patients [13]. Although AVF is the most ideal vascular pathway for MHD patients, its service life is not permanent: a 2014 study showed that the 1- and 2-year patency rates of AVF were 60% and 51%, respectively [14]; data from the 2016 DOPSS (Dialysis Outcomes and Practice Pattern Study) showed that the patency rate of autologous AVF1 was only 68% in the UK and relatively high in Europe (83%) [15]. In addition, a systematic review in 2016 showed that only 62-68% of AVF remained unobstructed after 1 year of use and dropped to 38-56% after 2 years [16]. The failure of AVF reduces the dialysis efficiency and quality of life of MHD patients and sometimes even threatens the lives of patients. This undoubtedly increases the pain and additional burden of patients. A survey found that the proportion of dialysis patients hospitalized due to AVF failure is as high as 20-25% [17, 18]. The functional status of arteriovenous fistula in patients with MHD is related to a variety of factors, including preoperative vascular condition, mode of operation, hypotension during dialysis, and inappropriate compression, which may lead to arteriovenous fistula stenosis or embolism [17]. In recent years, it has been found that the failure of arteriovenous fistula may be related to the general clinical data such as primary disease, sex, age, underlying disease, smoking history, hemoglobin, hematocrit, eosinophil, albumin, and coagulation related index. All of the above factors may increase the incidence of arteriovenous fistula stenosis or embolism [18]. Therefore, it is very important to maintain the good function of AVF in patients with MHD and to keep it unobstructed, and it is the direction of joint efforts of nephrology medical staff and patients [18].

RETRACTED

Richard et al.'s meta-analysis of 13 cohort studies showed that the elderly with head and neck AVF had a higher primary failure rate and a significant decrease in patency rate [19]. This may be related to the fact that the elderly are more likely to suffer from diabetes and peripheral vascular diseases, while studies by Garg et al. have indicated that diabetes is an independent risk factor for intima-media width in patients with renal disease, poor vascular conditions, and arterial intima-media thickening, which may lead to a higher proportion of arteriovenous fistula failure [20]. Other studies do not support that the decrease in the patency rate of arteriovenous fistulas in uremic patients is related to age [21]. In our study, logistic regression analysis uncovered that age was a risk factor for late failure of arteriovenous fistula in hemodialysis patients, which was consistent with the results of some researchers [20]. Anemia is a common complication in patients with ESRD, but with the use of erythropoietin (EPO) and iron, the level of hemoglobin in patients with MHD is significantly increased, and the level of HCT is also improved. Anemia symptoms of patients are better than before, but some studies have indicated that increasing the level of hemoglobin cannot improve the prognosis of patients with CKD; on the contrary, increased hemoglobin may increase the incidence of cardiovascular events and arteriovenous fistula embolism [22]. With the increase in hemoglobin and hematocrit, blood viscosity increases, resulting in an increased risk of arteriovenous fistula blockage. It has been indicated that the use of higher doses of erythropoietin is associated with vascular pathway thrombosis [22, 23]. This study indicated that the average hemoglobin level in the arteriovenous fistula failure group was higher than that in the patency group, which was consistent with the result of the Zhang study that the increase in HB was the cause of internal fistula obstruction [24]. Therefore, properly adjusting the dosage of erythropoietin in patients with ESRD anemia, slowly increasing the concentration of hemoglobin in patients with MHD, and maintaining it at an appropriate level have important clinical significance for the prevention of arteriovenous fistula embolism.

Eosinophils are present in human eosinophils, which are increased in hemodialysis patients due to exposure to various substances during HD [25]. It is reported that some materials can lead to eosinophil increase during dialysis, such as ethylene oxide and heparin, and heparin is often employed in hemodialysis [26]. Studies have indicated that there is a recognized clinical link between hypereosinophilic syndrome and thrombosis [27]. Previous studies have indicated that eosinophil cationic protein can enhance factor oxidation dependence and lose the anticoagulant activity of heparin, and some studies have indicated that the crystal structure of eosinophil basic protein specifically binds to heparin [28]. In our study, the proportion of eosinophils in the arteriovenous fistula failure group was significantly higher, and thrombosis was the most common cause of arteriovenous fistula failure. Therefore, this study supports the above results of the relationship between eosinophils and thromboembolism. The disorder of calcium and phosphorus metabolism is a common complication in patients with CKD. It is an important factor causing secondary hyperparathyroidism, calcium and phosphorus deposition, vitamin D metabolism disorder, and renal osteopathy. Studies have indicated that vascular calcium deposition in uremic patients is as active as bone deposition. In addition, the increase in calcium-phosphorus product can stimulate the proliferation of vascular smooth muscle cells, accelerate vascular calcification, increase the stiffness of arterial vessels, and worsen the function of vasomotor and vasomotor and is prone to vascular stenosis or occlusion [29–31]. In this study, the product of calcium and phosphorus in the arteriovenous fistula failure group was significantly higher compared to that in the control. Therefore, this study also confirmed that the increase in calcium-phosphorus product induced by calcium-phosphorus metabolism disorder in uremic patients increased the risk of arteriovenous fistula failure. It is worth mentioning that this study also has some shortcomings; for example, the number of cases included is not rich enough; meanwhile, this study is a retrospective study, and this study is a single-center study. Our conclusions need to be verified in a larger number of multicenter prospective studies in the future.

RETRACTED

Taken together, age, hemoglobin, hematocrit, and calcium-phosphorus product are independent risk factors for late failure of arteriovenous fistula in hemodialysis patients. The hemoglobin, eosinophil, platelet count, and hematocele in hemodialysis patients with late failure of arteriovenous fistula were higher. The indexes related to biochemistry, blood coagulation, and nutrition were significantly different from those without late failure of arteriovenous fistula. Thus, the risk of late failure of arteriovenous fistula can be predicted. In the meanwhile, attention should be paid to the patient's age, hemoglobin, hematocrit level, and calcium and phosphorus product, and preventive intervention measures should be taken in advance.

## Figures and Tables

**Figure 1:** HE staining results of late failure of arteriovenous fistula in hemodialysis patients. (a) Figure histological changes of the cephalic vein after (1) AVF, HE, 10 × 4. The intima showed obvious hyperplasia and thickening as indicated by the arrow. Eccentric, narrow lumen, mainly subendothelial fibrous connective tissue hyperplasia, interstitial osteoporosis, and edema, with myxoid degeneration. (b) Figure histological changes of the cephalic vein after (2) AVF, HE, 10 × 2. The arrows showed annular hyperplasia and thickening of the intima with obvious myxoid degeneration. (c) Figure histological changes of the cephalic vein after (3) AVF, HE, 10 × 4. The smooth muscle of media is diffusely proliferated, and the stroma is loose and swollen as indicated by the arrow. (d) Figure histological changes of the cephalic vein after (4) AVF, HE, 10 × 10. The media smooth muscle indicated by the arrow was oppressed and obviously atrophied and thinned.

**Table 1:** Comparison of two groups of general data ($\bar{x}\pm s,\;n\;\left(\%\right)$).

Group	Failure group (*n* = 35)	Patency group (*n* = 60)	*t*/*χ*^2^	*P*
Gender (male/female)	15/20	27/33	0.041	0.839
Age (years)	64.13 ± 2.11	60.85 ± 1.22	9.615	<0.01
Body mass index (kg/m^2^)	52.83 ± 3.12	54.67 ± 12.45	1.440	0.150
Smoking history	15 (42.86)	24 (40.00)	0.074	0.784
Diabetes	9 (25.71)	49 (81.67)	29.103	<0.01
High blood pressure	6 (17.14)	50 (83.33)	40.020	<0.01
Primary disease				
Uric acid nephropathy	0	2 (3.33)	1.191	0.274
Polycystic kidney	3 (8.57)	3 (5.00)	0.476	0.490
Chronic nephritis	13 (37.14)	32 (53.33)	2.324	0.127
Obstructive nephropathy	0	1 (1.67)	0.589	0.442

**Table 2:** Comparison of hemoglobin, eosinophil, platelet count, and hematocrit ($\bar{x}\pm s$).

Group	*N*	Hemoglobin (g/l)	Eosinophil (10^9^/l)	Platelet count (10^9^/l)	Hematocrit (%)
Patency group	60	93.83 ± 12.67	0.12 ± 0.12	218.93 ± 53.33	28.19 ± 5.22
Failure group	35	110.68 ± 23.45	0.38 ± 0.21	205.87 ± 34.66	34.91 ± 10.82
*t*		4.552	7.691	2.093	4.075
*P*		<0.01	<0.01	0.039	<0.01

**Table 3:** Comparison of biochemical and coagulation indexes between the two groups ($\bar{x}\pm s$).

Group	*N*	Calcium and phosphorus product (m^2^/dl^2^)	CRP (mg/l)	PT (s)	Fibrinogen	INR
Patency group	60	57.58 ± 12.35	5.18 ± 1.22	13.45 ± 1.45	466.93 ± 23.56	1.29 ± 0.12
Failure group	35	62.49 ± 10.33	7.18 ± 2.21	13.64 ± 1.23	413.74 ± 43.22	1.09 ± 0.12
*t*		2.232	5.691	0.650	7.773	7.836
*P*		0.028	<0.01	0.517	<0.01	<0.01

**Table 4:** Comparison of nutrition-related indexes between the two groups ($\bar{x}\pm s$).

Group	*N*	Plasma albumin (g/l)	Alkaline phosphatase (mmol/l)	Triglyceride (mmol/l)	Cholesterol (mmol/l)
Patency group	60	34.19 ± 8.22	84.94 ± 10.66	2.49 ± 0.67	4.18 ± 0.21
Failure group	35	37.44 ± 10.29	238.94 ± 12.56	1.39 ± 0.65	4.46 ± 0.54
*t*		2.713	63.560	7.803	3.588
*P*		<0.01	<0.01	<0.01	<0.01

RETRACTED

**Table 5:** Logistic regression analysis of risk factors for late failure of arteriovenous fistula in hemodialysis patients.

Variable	*b*	SE	Chi-square value	*P*	OR	95% CI for OR
Age	1.554	0.100	241.492	≤0.01	4.730	3.888-5.755
Diabetes history	1.456	1.310	1.235	0.266	4.289	0.329-55.902
High blood pressure	1.677	1.052	2.541	0.111	5.349	0.681-42.053
Uric acid nephropathy	1.455	1.115	1.703	0.192	4.284	0.482-38.107
Hemoglobin	0.953	0.032	886.923	≤0.01	2.593	2.436-2.761
Eosinophil	2.564	1.675	2.343	0.126	12.988	0.487-346.194
Hematocrit level	1.677	0.454	13.644	≤0.01	5.349	2.197-13.025
Calcium and phosphorus product	3.422	0.143	572.648	≤0.01	30.631	23.144-40.540
CRP horizontal	1.288	0.984	1.713	0.191	3.625	0.527-24.944
Fibrinogen	1.780	0.930	3.663	0.056	5.930	0.958-36.701
INR horizontal	2.320	1.340	2.998	0.083	10.176	0.736-140.668
Plasma protein	2.445	1.311	3.478	0.062	11.531	0.883-150.590
Alkaline phosphatase	1.453	0.993	2.141	0.143	4.276	0.611-29.943
Cholesterol level	0.567	0.332	2.917	0.088	1.763	0.920-3.379
Triglyceride	2.434	2.214	1.209	0.272	11.404	0.149-874.314

## Data Availability

No data were used to support this study.
